The article "Natural Cross Chlamydial Infection between Livestock and Free-Living Bird Species" was retracted in 2012. Reasons: fabricated or falsified data; misconduct by an author; ethical violations by an author; concerns about the data.

# Natural Cross Chlamydial Infection between Livestock and Free-Living Bird Species

**DOI:** 10.1371/journal.pone.0013512

**Published:** 2010-10-19

**Authors:** Jesús A. Lemus, Juan A. Fargallo, Pablo Vergara, Deseada Parejo, Eva Banda

**Affiliations:** 1 Departamento de Ecología Evolutiva, Museo Nacional de Ciencias Naturales (CSIC), Madrid, Spain; 2 School of Biological Sciences, Aberdeen Centre for Environmental Sustainability (ACES), University of Aberdeen, Aberdeen, United Kingdom; 3 Departmento de Ecología Funcional y Evolutiva, Estación Experimental de Zonas Áridas (CSIC), Almería, Spain; 4 Oficina de Especies Migratorias, Ministerio de Medio Ambiente y Medio Rural y Marino, Madrid, Spain; Technical University Munich, Germany

## Abstract

The study of cross-species pathogen transmission is essential to understanding the epizootiology and epidemiology of infectious diseases. Avian chlamydiosis is a zoonotic disease whose effects have been mainly investigated in humans, poultry and pet birds. It has been suggested that wild bird species play an important role as reservoirs for this disease. During a comparative health status survey in common (*Falco tinnunculus*) and lesser (*Falco naumanni*) kestrel populations in Spain, acute gammapathies were detected. We investigated whether gammapathies were associated with *Chlamydiaceae* infections. We recorded the prevalence of different *Chlamydiaceae* species in nestlings of both kestrel species in three different study areas. *Chlamydophila psittaci* serovar I (or *Chlamydophila abortus*), an ovine pathogen causing late-term abortions, was isolated from all the nestlings of both kestrel species in one of the three studied areas, a location with extensive ovine livestock enzootic of this atypical bacteria and where gammapathies were recorded. Serovar and genetic cluster analysis of the kestrel isolates from this area showed serovars A and C and the genetic cluster 1 and were different than those isolated from the other two areas. The serovar I in this area was also isolated from sheep abortions, sheep faeces, sheep stable dust, nest dust of both kestrel species, carrion beetles (*Silphidae*) and Orthoptera. This fact was not observed in other areas. In addition, we found kestrels to be infected by *Chlamydia suis* and *Chlamydia muridarum*, the first time these have been detected in birds. Our study evidences a pathogen transmission from ruminants to birds, highlighting the importance of this potential and unexplored mechanism of infection in an ecological context. On the other hand, it is reported a pathogen transmission from livestock to wildlife, revealing new and scarcely investigated anthropogenic threats for wild and endangered species.

## Introduction

Cross-species infection is a major cause of emerging infectious diseases [1]-[3]. The economic influence of the animal industry has promoted many investigations regarding the potential of wildlife as a reservoir of cattle and poultry diseases [4], [5]. On the contrary, little is known about the role of domestic species as infectious agents causing diseases in wildlife [5], [6].

Avian chlamydiosis is a well-known human disease caused by the bacterium *Chlamydophila psittaci* [7]–[10] and contracted from poultry and wild birds, although pet bird (mainly parrots) are still considered the primary cause [11], [12]. In the wild, isolates have been reported from more than 460 avian species [9] as well as from some mammals, such as hares and muskrats [12], [13]. In birds it is often systemic and infections can be unapparent, severe, acute or chronic with intermittent shedding [12]. *Chlamydophila abortus* (also identified as *Chlamydophila psittaci* serovar I) is an abortogenic pathogen in ruminants rarely found in birds [14]. Factors leading to different degrees of symptomatology of this disease may be both internal, such as immune capacity, and external, such as stress [15], [16]. Indeed, adults more often have non-symptomatic infections while young birds frequently have acute disease, probably because adults are able to develop a better immunity response than young birds [15]–[17]. Additionally, stress will commonly trigger the onset of severe symptoms, resulting in rapid deterioration and death [18], [19].

Death outbreaks due to chlamydiosis can be found in wild bird species and are presumed to be due to infection with a strain uncommon to the host or due to secondary infections [11]. Chlamydiosis has been reported to be transferred by translocation of birds of prey, to spread during falconry bird flight or to spread across countries by migratory species [20], [21]. It has also been noted that colonially nesting birds are more likely to spread disease during reproduction than solitary breeders [22]–[24].

Chlamydiosis transmission from mammals to birds has been scarcely investigated, even with the knowledge that parenterally inoculated, polyarthritis-producing chlamydiae of ovine origin affected the leg joints of turkeys, and abortion-producing chlamydiae of ovine origin was infectious for pigeons and fatal for sparrows. Also, several species of small wild birds when inoculated perorally with *C. psittaci* of turkey origin, seroconverted (36%) and shed the organism (79%) [9]. In this same review, authors also indicated that their aim was to determine whether strains of *C. psittaci* from domesticated ruminants would infect, multiply in, or be shed by these wild birds, indicating whether or not these species of birds are natural hosts or biologic vectors of these strains. However, considering the heterogeneity of the chlamydial species, certain birds may harbour strains that are associated with naturally occurring infections in some animals. The results are also additional evidence of the more restricted host range of mammalian *Chlamydia* species when compared with avian isolates.

In this article we present the results of an episode of clinical chlamydiosis in common kestrels (*Falco tinnunculus*) and lesser kestrels (*F. naumanni*). During a study about kestrel health status [25], most of the birds in a given area showed a marked gammapathy in the protein electrophoresis pattern. We explored the origin of this abnormality. Gammapathies are well-documented as specific clinical laboratory tools for the study of several infections, including *Salmonella* and *Chlamydophila psittaci* [15], [26]. We show the results of serology, PCR studies and the serovar and genetic clusters of the isolated *Chlamydophila psittaci* samples, and we explore the possibility of *Chlamydophila psittaci* cross-species transmission. Additionally, other chlamydial species such as *Chlamydia muridarum* and *Chlamydia suis* were tested in spite of the fact that they have not shown to be of major interest in veterinary medicine or as cross-species transmission pathogens. *Chlamydia muridarum* is a rodent pathogen, especially of laboratory mice and hamsters, causing respiratory disease. No records have been published about its incidence in wild rodents or birds. *Chlamydia suis*, on the other hand, is a swine pathogen that causes important economic losses in intensive swine production due to digestive disease, and is extremely resistant to most antibiotics. There is no report about its incidence in extensive swine or in birds.

There is some controversy in Chlamydiaceae taxonomy [7], [8], [27], [28], and especially in the *psittaci* serovars involved in livestock diseases [28]. We followed the taxonomy proposed by Schiller et al (2004) [28].

## Results

Protein electrophoresis showed that both kestrel species from LL showed higher levels of γ-globulins than kestrels from CA and LM, being this difference statistically significant (GLMM, *F*_2,65_ = 47.73, *P*<0.001, Fig. 1). Lesser kestrels showed higher values than common kestrels (GLMM, *F*_1,65_ = 15.47,*P*<0.001, Fig. 2). This was due to the between-species difference found in LL while no between-species differences were found in CA and LM. This resulted in a significant species x area interaction (GLMM, *F*_2,65_ = 23.89, *P*<0.001, Fig. 2). In Figure 3 the protein electrophoresis profiles in LL kestrels are represented showing a standard profile and the detected gammapathies.

**Figure 1:** Between-area differences in kestrel gammaglobulin levels. Differences in gammaglobulin levels (percentage of total proteins) between the three study areas for both Eurasian and Lesser kestrels. Interaction between species and study area is statistically significant.

**Figure 2:** Gammaglobulin levels in infected and uninfected kestrels. Differences in gammaglobulin levels (percentage of total proteins) between kestrels uninfected and infected by *Chlamydophila abortus* (*Chlamydophila psittaci* serovar I). The interaction between infection and species is statistically significant.

**Figure 3:** Protein electrophoretic pattern. A) Protein electrophoretic profile showing a typical gammapathy found in kestrel individuals infected by *Chlamydophila abortus* (*Chlamydophila psittaci* serovar I). B) Normal kestrel protein electrophoretic profile.

*Chlamydophila abortus* (*C.p.* serovar I) was the most prevalent of the three species found in kestrel populations (12.6%), followed by *Chlamydia suis* (5.7%) with the prevalence of *Chlamydia muridarum* the lowest (3.8%). All individuals infected by *Chlamydia suis* were also infected by *Chlamydophila abortus*, while none of the individuals infected by *C. muridarum* were found to be infected by any other *Chlamydiaceae* species. In order to explore gammapathies associated with a given *Chlamydiaceae* species we excluded from the analyses individuals infected with the other two species, thus comparing infected vs. uninfected individuals. Gammapathies in kestrels were found to be associated with *Chlamydophila abortus* (*C.p.* serovar I) infection (Table 1), showing significantly higher levels of immunoglobulins in blood in infected compared to uninfected individuals (Fig. 3). The model also showed significant differences between kestrel species and significant infection x species interaction (Table 1, Fig. 3). Similar results were found for *Chlamydia suis* infection (Table 1). However, note that all of these individuals were also infected by *Chlamydophila abortus*, for which reason we could not separate the effect of both Chlamydiaceae species. Gammapathies in kestrels were not found to be associated with *Chlamydia muridarum* (Table 1).

**Table 1:** Effects of kestrel species and *Chlamydiaceae* infection on immunoglobulin levels.

	*F*	*d.f.*	*P*
***Chlamydophila abortus***			
Infection	29.62	1,59	<0.001
Species	39.14	1,59	<0.001
Infection * species	42.09	1,59	<0.001
***Chlamydia muridarum***			
Infection	0.25	1,62	0.624
Species	0.13	1,62	0.653
Infection * species	0.03	1,62	0.877
***Chlamydia suis***			
Infection	6.21	1,57	0.004
Species	5.43	1,57	0.023
Infection * species	6.40	1,57	0.014

Results of general linear mixed models (GLMM) in which immunoglobulin levels are included as a response variable and infection (infected vs. uninfected) and kestrel species are fixed factors. Between-factor interaction is also shown.

Serology analyses showed that all nestlings from LL had *Chlamydophila psittaci* (*C.p*.) antibodies, while only a small proportion of kestrels from LM and none from CA had these antibodies (Table 2). Between-area differences were significant for both common (GENMOD, χ^2^ = 51.18, *d.f.* = 2, *P*<0.001) and lesser (GENMOD, χ^2^ = 44.46, *d.f.* = 2, *P*<0.001) kestrels. No other antibodies were found during the serology evaluation. Due to the results obtained from the samples, we prepared a serovar and cluster double blind study in order to establish the *Chlamydophila* origin.

**Table 2:** Prevalence of *Chlamydiaceae* species.

	*Falco tinnunculus*			*Falco naumanni*		
	*CA* (*n* = 19)	*LM* (*n* = 8)	*LL* (*n* = 17)	*CA* (*n = 6*)	*LM (n = 28*)	*LL* (*n* = 13)
*Chlamydophila psittaci* antibody serology	0% (0)a	25% (2)b	100% (17)c	0% (0)a	7.1% (2)a	100% (13)b
Classical *Chlamydophila psittaci* PCR	26.3% (5)a	37.5% (3)a	100% (17)b	33.3% (2)a	25% (7)a	100% (13)b
Real time *Chlamydophila psittaci* PCR	26.3% (5)a	37.5% (3)a	100% (17)b	33.3% (2)a	25% (7)a	100%(13)b
*Chlamydophila abortus* (*Chlamydophila psittaci* serovar I)	0% (0)a	0% (0)a	64.7% (11)b	0% (0)a	0 % (0)a	61.5% (8)b
*Chlamydophila abortus* MLST	0% (0)a	0% (0)a	64.7% (11)b	0% (0)a	0 % (0)a	61.5% (8)b
*Chlamydia muridarum*	5.3% (1)a	0% (0)a	0% (0)a	16.7% (1)	0 % (0)	(0)
*Chlamydia suis*	0% (0)a	0% (0)a	35.3% (6)b	0% (0)ac	0 % (0)a	23.0% (3)bc

Prevalence of *Chlamydiaceae* species and strains isolated from both kestrel species in different areas. Prevalence is expressed as percentage of infected individuals. Numbers in brackets represent infected individuals. Different letters indicate between-area significant differences as resulted from between-group contrasts in GENMOD procedure.

First, we performed a classical *Chlamydophila psittaci* PCR *C.p.* and real time PCRs. Both PCRs showed the same result, *C.p.* being identified in all individuals from LL, while only a small proportion of kestrels showed *C.p.* in the other two areas (Table 2). The difference was significant for both kestrel species (GENMOD, both *P*<0.001)

We found that a proportion of kestrels from LL, but no kestrels from the other two areas had antibodies for *C. abortus* (*C.p.* serovar I) and *C. suis*. The between-area differences were significant for *C. abortus* and *C. suis* in both kestrel species (GENMOD, all *P*<0.017), while no between-area differences were found in *C. muridarum* in any of the kestrel species (GENMOD, both *P>*0.43). MLST analysis showed the same results observed with PCRs (Table 2).

Serovar characterization indicated that both kestrel species from LL showed positive tests for serovars A and C of *C.p.*, while kestrels from CA and LM were positive for serovars F and G (Table 3).

**Table 3:** *Chlamydophila psittaci filiation.*

	*Falco tinnunculus*			*Falco naumanni*		
	Campo Azálvaro (CA)	Los Monegros (LM)	Los Llanos (LL)	Campo Azálvaro (CA)	Los Monegros (LM)	Los Llanos (LL)
Serovar						
A	-	-	2	-	-	6
B	-	-	-	-	-	-
C	-	-	16	-	-	5
D	-	-	-	-	-	-
E	-	-	-	-	-	-
F	1	5	-	2	13	-
G	7	3	-	4	1	-
Clusters						
I	-	-	13	2	2	7
II	-	5	-	3	10	-
III	3	3	5	1	2	4
IV	5	-	-	-	-	-

*Chlamydophila psittaci* filiation based in serovars and genetic clusters (ordered following avian phylogenetic origin) of the different kestrel isolates from the three sampled locations.

Genetic cluster analyses for *C.p.* indicated that kestrel samples from LL were located mainly in cluster I with few samples belonging to cluster III. Lesser kestrels from CA and LM populations mainly “showed clusters” of type II and few of type I and III. Finally, common kestrels from CA and LM populations only showed clusters of type II and III (see Table 3).

In LL, *C. abortus* (*C.p.* serovar I) was found in all the possible sources explored: sheep abortions, sheep faeces, sheep stable dust, nest dust of both kestrel species, carrion beetles (*Silphidae*) and Orthoptera (Table 4). In LM, it was found in lower proportions in sheep stable dust. *C.p.* was also found in low proportion in samples of stable dust, lesser kestrel nest dust and Orthoptera. In CA, kestrels breed in nest boxes and old buildings, for which reason only Orthoptera invertebrates were checked. We did not find *Chlamydophila* in these prey species from this locality.

**Table 4:** Presence of *Chlamydophila* in kestrel environment.

	Los Llanos (LL)			Campo Azálvaro (CA)			Los Monegros (LM)		
	*N*	*C psittaci*	*C abortus (C psittaci serovar I)*	*n*	*C psittaci*	*C abortus (C psittaci serovar I)*	*n*	*C psittaci*	*C abortus (C psittaci serovar I)*
Sheep abortions	16	0	16	a	-	-	3	0	0
Sheep faeces (Facilities)	26	0	9	-	-	-	14	0	0
Sheep stable dust (Facilities)	14	0	7	-	-	-	12	1	2
Eurasian kestrel nest dust	25	0	9	b	-	-	10	0	0
Lesser kestrel nest dust	22	0	15	c	-	-	16	7	0
Carrion beetles	8	0	4	0	-	-	4	0	0
Grasshoppers/locust/crickets	60	0	18	60	0	0	60	1	0

Presence of *Chlamydophila psittaci* and *C. abortus* (*C. psittaci* serovar I) in different potential sources of infection for kestrel species.

a No sheep presence in the area.

b Nests in nest-boxes.

c Nest material was not collected.

## Discussion

Exploring the health status of common and lesser kestrel populations from three different locations we detected gammapathies in individuals of both species in one of the locations (LL). This gammapathy was found to be associated with infections of *Chlamydophila abortus* (*C. psittaci* serovar I). In this same area a *Chlamydophila* outbreak was observed in sheep, sheep facilities and also in insects, suggesting a cross *Chlamydophila* infection between livestock and wild insect and bird species.

Chlamydiosis diagnosis is difficult, because there are many false negatives due to the absence of immunological reaction. In our case, common and lesser kestrel nestlings from LL showed a response to infection in protein electrophoresis and serology that was not observed in kestrels from the other two areas. Within the LL area, lesser kestrels showed stronger gammapathies (higher percentage of immunoglobulins) than common kestrels. Between-species differences can be promoted by differences in diet, as lesser kestrels are more insectivorous, thus more prone to ingesting carrion beetles and Orthoptera carrying *C.p.* serovar I. Furthermore, lesser kestrels tend to use sheep stables as breeding sites in a higher proportion than common kestrels, hence being more exposed to inhaling *Chlamydophila* fomites, such as dust.

In this study we have tried all diagnostic procedures with the exception of culture. Detection by PCR only isolates genetic material, not pathogens, but allows the detection of Chlamydiaceae exposure. When combining Chlamydiaceae with the determination of pathogen antibodies we can clearly detect those individuals that are clinically infected.

*Chlamydophila psittaci* is ubiquitous and causes many different diseases and prognoses in birds, and is more aggressive in nestlings [29]. In a previous paper we showed that those kestrels from LL were in poorer condition when compared to CA and LM individuals [25].

Serovar characterization and genetic clusters indicate zone differentiation in the serovars affecting kestrels. While LL typical serovars are A and C of *C.p.*, kestrels from CA and LM were positive for serovars F and G (Table 3), the serovars typical of raptors [9], [27]. Few wildlife studies have described *C.p.* clusters. Our study also indicates this zone differentiation in *C.p.* clusters. Isolates from LL were located mainly in cluster I with few samples belonging to cluster III. Lesser kestrel isolates from CA and LM populations were mainly clustered in type II and few of the type I and III. Finally, common kestrels from CA and LM populations only showed clusters of type II and III. Together, these results indicate the origin of all isolates and permit the linkage of isolates to their original host. With the exception of the ruminant-hosted *C.p*. serovar I, the remaining *Chlamydophila* isolated from kestrels were avian-hosted *Chlamydophila*. Serovar A (found in LL) is naturally hosted by psittacines, columbids and several corvids [9], [27], while serovar C is naturally hosted by storks [9], [27]. Raptors are not natural hosts for either serovar. On the contrary, kestrels from CA and LM were infected with typical F or G serovars that are only susceptible to disease in case of immunological disruption, since these serovars are considered to be moderately pathogenic in their natural hosts [9], [27].

Enzootic abortion (the denomination of *C.p*. serovar I in sheep) is endemic in Spanish locations, including the Extremadura region where the *Chlamydophila* outbreak was found [30]. Abortions and mothers remain uncontrolled in the field with no assistance. We have identified potential infectious agents that can act through the two known *Chlamydophila* transmission routes: ingestion and inhalation. Invertebrates can be infected by direct consumption of sheep abortions, carcasses and faeces. Apart from these routes, vertebrates, as in the case of kestrels, can also be infected through the ingestion of infected insects. The presence of *C. p.* in dust from sheep facilities (also in kestrel nests) suggests that both vertebrates and invertebrates can contract the disease through inhalation in the surroundings of sheep stables. Measures including 1) vaccination [31] of all the sheep at risk or in enzootic areas and 2) increasing the frequency of health controls should be mandatory to minimize the risk of transmission to wildlife. To our knowledge this is the first study in which *Chlamydophila psittaci* is detected in livestock remains and in the environment. This isolation reflects the infective potential of this pathogen and the environmental dependence of prophylactic measures in order to avoid cross-species transmission. It is important to be aware of the potential of zoonotic transmission of *C. psittaci* from poultry to men [32]–[34], and also the zoonotic potential to pregnant women [35].

Similarly, *Chlamydia suis* and *C. muridarum* have never been recorded in birds. They typically appear in swine and rodents, respectively [12]. In principle, this suggests two more cases of cross-species pathogen transmission found in this study, which would be expected to provoke a conspicuous immune reaction. However, we have only actually detected the genetic material of these two species, because no antibody reactions have occurred in the serology panel. This was observed in the case of *C. suis*. However, due to the fact that individuals infected by *C. suis* were infected by *Chlamydophila abortus* as well, we could not disentangle its true effect on immunoglobulin levels. In the case of *C. muridarum* we did not detect gammapathies in infected individuals. The paucity of knowledge about *Chlamydiaceae* pathology in wildlife makes it difficult to explain this lack of immunological reaction. One possibility is that we are only measuring one component of the immune system, and that other immunological branches, such as a cell-mediated immune response, could be acting without our detection. A second possibility is that *C. muridarum* could be a common pathogen in kestrels, as they usually prey on rodents. In this sense, our study highlights the interest of investigating this aspect in future studies.

The lesser kestrel is considered as a “Vulnerable” species throughout its range (www.iucnredlist.org, 25). Farmlands and grasslands are the most common habitats for this species [36]. Extremadura possesses up to 25% of the lesser kestrel Spanish population and its numbers have shown a positive trend over the last several years [37]. The common kestrel, on the other hand, is the most common diurnal raptor species in Spain, however with negative population trends in Europe [38]. The changes in land-use practices (agricultural intensification and pesticide use) and direct persecution have traditionally been the causes proposed to explain population declines in both kestrel species [37]–[40]. However, other problems more subtle to identify, such as infectious disease episodes, call into question the conservation efforts, especially those devoted to the lesser kestrel. Epizooties can operate in wild species causing population declines at a local scale [41]–[43]. Wildlife populations are immunologically prepared for many of the pathogens in the environment, but changes in the serovars usually imply mortality episodes [3], [4], [6]. Our study emphasizes the necessity of wildlife veterinary controls as useful tools for conservation plans and detection of risks in wild species.

## Materials and Methods

### Samples examined

We tested for *Chlamydophila psittaci* in a total of 91 common (n = 44) and lesser (n = 47) kestrel nests present in three study areas located in Los Llanos (Cáceres province, 39° 28′ N, 6° 22′ W), Campo Azálvaro (Segovia province, 40° 40′ N, 4° 20′ W) and Los Monegros (Zaragoza province, 41° 20′ N, 0° 11′ W). The three locations are subjected to high extensive livestock pressure, with extensive ovine livestock in Los Llanos (LL) and Los Monegros (LM) and extensive bovine livestock in Campo Azálvaro (CA); see Vergara et al. (2008) [25] for more study area characteristics. Ovine livestock receive no veterinary interference except legal controls in LL, and receive some veterinary assistance and prophylactic treatments in LM. Sample size for each kestrel species and area is shown in Table 2. One chick per nest in each kestrel species was randomly selected for blood samples.

All the nestlings were sampled at about three weeks old. One ml of blood was taken from the brachial vein, centrifuged and the pellet was separated from plasma and both were frozen until analyses.

### Protein electrophoresis

As a part of the health status design, protein electrophoresis was performed in all checked specimens. Plasma protein electrophoresis fractions were run on commercial agarose gels (Hydragel Protein (E), Sebia Hispania S.A., Barcelona, Spain) using a semi-automated Hydrasys System (Sebia Hispania S.A., Barcelona, Spain) with manufacturer's reagents to determine the concentration of albumin and globulins (α, β and γ-globulins) in percent, that were used in the analyses. Total plasma proteins were determined by the Biuret method [44]. Total plasma protein concentrations (g/dl), which were also used in the analyses, were calculated by the multiplication of each protein fraction with the total protein value.

### *Chlamydophila psittaci* serology

A serology panel that included *Salmonella* and *Chlamydophila psittaci* serology was performed using plasma samples. A whole blood-plate agglutination test was used to detect the *Salmonella* antigen presence Difco (TM) *Salmonella* O Group B Antigen (1-4-5-13) (Becton Dickinson and Company, Maryland, USA). The test was conducted by using the manufacturer's standard instructions [45]. *Chlamydophila psittaci* antibodies were determined by using Rida-Screen antibody ELISA (R-Biopharm, Darmstadt, Germany)

### *Chlamydophila psittaci* PCR, real time PCR and *Chlamydophila abortus* (*Chlamydophila psittaci* serovar I) PCR

Blood PCRs were performed following Hewinson et al, 1997, for conventional PCR for *Chlamydophila psittaci*, Sachse et al, 2009, for real time PCR *for Chlamydophila psittaci*, and Laroucau et al, 2001 were used to *Chlamydophila abortus* conventional PCR [46]–[48]. We have considered *Chlamydophila psittaci* serovar I as *Chlamydophila abortus*, following Kaleta & Taday (2003) [9] and Schiller et al. (2004) [28]. This technique has been demonstrated to be successful when showing pathogen exposure in common and lesser kestrels [49].

Due to the presence of extensive livestock in the area, and the occurrence of enzootic chlamydial abortion, we also performed a chlamydial serovar characterization to establish the serovar involved in the epizootic episode. In addition, we also obtained the genetic cluster of the same isolates according to Chahota et al, 2006 [14]. We explored the presence of *Chlamydia* species, *Chlamydia suis and Chlamydia muridarum.* For *Chlamydia suis* we used the specification of Laroucau et al, 2001, and Robertson et al, 2009 [48], [50] whilst for *C. muridarum* we used the specifications of Pantchev et al and Robertson et al, 2009 [50], [51]

### Serovar characterization

For serovar characterization the isolates were either grown directly in Buffalo green monkey (BGM) cells or in 6-day-old specific pathogen-free embryonated chicken eggs as is indicated in Vanrompay et al, 1993 [27]. The six serovar- specific MAbs were designated VS-1 (serovar A specific; psittacine group), CP3 (serovar B specific; pigeon I group), GR-9 (serovar C specific; duck group), NJ-1 (serovar D specific; turkey group), MP (serovar E specific; pigeon II group), NJ-1D3 (serovar F) and serovar G [52]. The microimmunofluorescence test was also performed following Vanrompay et al. (1993) [27].

### *Chlamydophila* genetic diversity

Genetic diversity and epizootiology of *Chlamydophila psittaci* was based on the VD2 region of the *ompA* gene. DNA was extracted, a nested PCR was performed followed by cloning of the PCR product and sequencing [14]. The sequence analyses were performed following Chahota et al. (2006) [14].

We also tested for *Chlamydophila psittaci* type I in sheep abortions, sheep faeces, sheep stable dust, kestrel nest dust, necrophilous beetles and orthoptera (grasshoppers, locusts, crickets) in the study areas. Beetles and orthoptera are common prey species of common and lesser kestrels in Spain [36], [53]. Arthropods were collected close to nests (50 m away from carcasses in the case of beetles and 200 m away from nests in the case of orthoptera), and were euthanized by congelation.

Sheep abortion samples were processed following Schiller et al, 2004 [28], whilst sheep faeces and dust preparation was performed following Tanaka et al, 2005 [54], and arthropods were prepared by homogenization [55].

### *Chlamydophila abortus* MLST analysis

Because of the difficulty to discriminate between *C. psittaci* and *C. abortus* and not possible on the basis of the major outer membrane protein A, we additionally carried out a. MLST analyses as described by Pannekoek et al.(http://www.pubmlst.org/chlamydiales).

### Statistical procedures

Nestlings share genes and environments within the nest for which reason these cannot be considered independent samples. We attempted to analyse between-location and between-species differences in nestling infection (infected vs. uninfected) by using Generalized Mixed Models, in which the nest was included as a random factor and species as a fixed factor. This procedure avoids pseudoreplication considering the nestling as the sampling unit. Due to the fact that some chlamydial isolates where absent in some locations our data were unbalanced and most of the models did not converge. For this reason we randomly selected one nestling from each nest and analysed frequencies of infection in different locations and species by using GENMOD procedure with logit link function and binomial distribution in SAS statistical software (SAS 9.0, 2002, Institute Inc., Cary, NC, USA). Differences in protein electrophoresis between kestrel species and populations were analysed using General Linear Mixed Models with GLMM procedure in. The percentage of γ-globulins was arcsine transformed. Nest was included in the model as a random factor and location and species as fixed factors.

### Ethics Statement

Our study followed ethical guidelines proposed for the Spanish Royal Decree 1205/2005 about the protection of animals used in experiments and scientific research and was approved by the Spanish Ministry of Science and Innovation (CGL2007-61395/BOS).
